The article "Effects of Dexmedetomidine on Postoperative Pain and Recovery Time in Obese Patients" was retracted in 2023. Reasons: suspected computer-generated content; unreliable results or conclusions; concerns about the data; concerns about the results or conclusions.

# Effects of Dexmedetomidine on Postoperative Pain and Recovery Time in Obese Patients

**DOI:** 10.1155/2022/9715704

**Published:** 2022-09-28

**Authors:** Qian Zhang, Zhaojian Zhang, Bing Wang, Chao Zhao, Yuedan Xu

**Affiliations:** Department of Anesthesiology, The First People's Hospital of Lianyungang, No. 182, Tongguan North Road, Lianyungang, 222000 Jiangsu, China

## Abstract

**Objective:**

The objective of this study is to investigate the effect of dexmedetomidine on postoperative pain and recovery time in obese patients.

**Methods:**

A total of 100 obese patients with body mass index (BMI) ≥ 30 kg/m^2^ who underwent laparoscopic sleeve gastrectomy under general anesthesia in our hospital from January 2019 to December 2021 were included and assigned into DEX group (dexmedetomidine group) and NS group (normal saline group). The bariatric surgery patients who were given normal saline pump were the NS group (*n* = 50), and the bariatric surgery patients who were given the dexmedetomidine pump were the DEX group (*n* = 50). The patients in the DEX group were given continuous intravenous infusion of dexmedetomidine before, during, and after induction of anesthesia at a dose of 0.4 *μ*g. kg-1. h-1, 0.4 *μ*g·kg-1. h-1, 0.2 *μ*g·kg-1. h-1, respectively. The NS group was infused with the same volume of normal saline for the same time. The two groups of patients were treated with the same anesthesia induction and maintenance program. By comparing the operation, anesthesia, postoperative extubation, and recovery time of the two groups of patients, the effect of dexmedetomidine on the postoperative recovery time of obese patients was analyzed. Visual analogue scale (VAS) and adverse reactions were compared to analyze the effect of dexmedetomidine on postoperative pain in obese patients.

**Results:**

The operation, anesthesia, postoperative extubation, and recovery time of the DEX group were significantly lower than those of the NS group, whereas the VAS and adverse reactions were significantly lower than those in the NS group (*P* < 0.05).

**Conclusion:**

An appropriate dose of dexmedetomidine in bariatric surgery for morbidly obese patients can effectively shorten the recovery time and extubation time of patients, reduce postoperative pain and the incidence of adverse reactions, and is worthy of clinical application. Dexmedetomidine 2 *μ*g/kg has promising anesthesia benefits in bariatric surgery of obese patients, can provide favorable analgesia and quality of recovery, help reduce the degree of stress response of patients, and does not increase the risk of adverse events. However, this study has certain limitations, so physicians should tailor the dosage according to the patient's physical condition in clinical practice.

The article "Effects of Dexmedetomidine on Postoperative Pain and Recovery Time in Obese Patients" was retracted in 2023. Reasons: suspected computer-generated content; unreliable results or conclusions; concerns about the data; concerns about the results or conclusions.

## 1. Introduction

Obesity is a chronic metabolic disease that is an abnormal or excessive fat accumulation affecting human health as defined by the World Health Organization (WHO) [1]. The change of lifestyle and the improvement of living standards have led obesity to become one of the serious public health problems worldwide. Obesity is also complicated by sleep apnea, impaired reproductive function, hypertension, diabetes, cardiovascular and cerebrovascular diseases, osteoarthritis, and even tumor diseases, posing a serious threat to the physical and mental health of patients [2, 3]. The mainstays include controlling diet, strengthening exercise, and drug therapy, yet they are not available to all obese patients. For patients with severe simple obesity and serious complications, surgery is the ultimate method of obesity treatment [4]. Multiple studies with large samples have shown that the most effective modality for the treatment of obesity and its associated diseases is bariatric surgery.

Laparoscopic sleeve gastrectomy, which is widely used today, can effectively control the synthesis of hepatic glucose and relieve fatty liver, hypertension, and lipid metabolism disorders in patients [5]. And laparoscopic bariatric surgery has raised considerable concern due to its merits of less trauma, short operation time, persistent advancement of surgical methods, rapid postoperative recovery, high safety, and feasibility to the two major problems of obese patients (i.e., the difficulty of surgical field exposure and postoperative fat liquefaction). However, this surgical treatment requires intraoperative CO_2_ pneumoperitoneum. Due to the reduced lung compliance, increased diaphragm muscle, and potential respiratory dysfunction in obese patients, many patients often have psychological stress reactions such as restlessness, depression, and tension after entering the postanesthesia care unit (PACU), which immensely compromises the surgical treatment outcomes [6]. Therefore, it is vital to choose safe, effective, and appropriate doses of sedative and analgesic drugs during the operation to facilitate the postoperative recovery of patients.

Dexmedetomidine (Dex) is a new type of *α*2 adrenergic receptor agonist and it can selectively bind to *α*2, *α*1, adrenergic receptors. The locus coeruleus of the brainstem can participate in the transmission of sympathetic nerve signals from the center to the periphery and is the area with the most dense *α*2 receptors in the brain. Dexmedetomidine can act on *α*2 adrenergic receptors in the locus coeruleus of the brainstem, resulting in sedative, hypnotic, and anxiolytic effects. Studies have shown that the use of dexmedetomidine, compared with other sedative drugs, can lead to an awakening effect from sedative state. As a result, the patients can more cooperate with the doctor's instructions, and it can also reduce the concentration of catecholamines in plasma and inhibit the release of norepinephrine, thereby reducing the stress response. Dexmedetomidine is different from traditional sedative drugs such as propofol. The dexmedetomidine dominantly acts on the key part of the brain responsible for regulating sleep and wakefulness, i.e., the blue spotted areas of the brainstem, and its sedative effect does not require GABA pathway to work [7, 8]. To the end, this study intends to compare the effects of saline and Dex on postoperative pain and recovery time in obese patients undergoing bariatric surgery.

The article "Effects of Dexmedetomidine on Postoperative Pain and Recovery Time in Obese Patients" was retracted in 2023. Reasons: suspected computer-generated content; unreliable results or conclusions; concerns about the data; concerns about the results or conclusions.

## 2. Materials and Methods

### 2.1. Baseline Data

A total of 100 obese patients with body mass index (BMI) ≥ 30 kg/m2 who underwent laparoscopic sleeve gastrectomy under general anesthesia in our hospital from January 2019 to December 2021 were selected and assigned into DEX group (dexmedetomidine group) and NS group (saline group) according to a randomization calculator (http://www.randomization.com). The bariatric surgery patients who were given normal saline pump were the NS group (*n* = 50), and the bariatric surgery patients who were given the dexmedetomidine pump were the DEX group (*n* = 50). The patients in the DEX group were given continuous intravenous infusion of dexmedetomidine before, during, and after induction of anesthesia at a dose of 0.4 *μ*g. kg-1. h-1, 0.4 *μ*g·kg-1. h-1, 0.2 *μ*g·kg-1. h-1, respectively. The NS group was infused with the same volume of normal saline. The two groups of patients were treated with the same anesthesia induction and maintenance program.

#### 2.1.1. Sample Size Estimation

We use the improvement of MMSE scores as the main effect indicators to estimate the sample size. Sample size calculations are performed to determine the number of participants needed to detect effect sizes. About 30-50 individuals per group will be calculated according to the formula. With a type I error of 5% (*α* = 0.05) and 90% power (*β* = 0.10).

#### 2.1.2. Ethical Considerations

Patients who were scheduled to have an SCS trial were approached and given a Patient Information Sheet to take home to read. Informed consent was obtained from suitable patients after a reasonable period by one of the principal investigators or delegated individuals at each site following International Conference on Harmonization/Good Clinical Practice (ICH/GCP) guidelines. The study was approved by the First People's Hospital of Lianyungang. The trial was conducted and reported in accordance with CONSORT guidelines.

The article "Effects of Dexmedetomidine on Postoperative Pain and Recovery Time in Obese Patients" was retracted in 2023. Reasons: suspected computer-generated content; unreliable results or conclusions; concerns about the data; concerns about the results or conclusions.

### 2.2. Inclusion and Exclusion Criteria

#### 2.2.1. Inclusion Criteria

The inclusion criteria are the following: (1) with surgical indications, (2) with stable vital signs, (3) without previous mental illness and cognitive impairment, (4) American Society of Anesthesiologists (ASA) I-III, and (5) with complete clinical data.

#### 2.2.2. Exclusion Criteria

The exclusion criteria are the following: (1) patients with contraindications to surgery and anesthesia, (2) patients with severe liver and kidney dysfunction, (3) patients with cognitive impairment or mental illness, (4) those who use sedative and analgesics for a long time, (5) those who prepare for pregnancy within 2 years after surgery, (6) those who are allergic to dexmedetomidine or other ingredients in the drug, (7) concomitantly use of a monoamine oxidase inhibitor or within 2 weeks after stopping, (8) long-term heavy drinkers, (9) patients with anatomical variation and difficulty in endotracheal intubation, and (10) those with communication barriers and unable to cooperate with postoperative follow-up.

### 2.3. Methods

#### 2.3.1. Anesthesia Induction

All patients were routinely fasted for 8 hours and water-forbidden for 4 hours preoperatively without preoperative medication. After the patient entered the operating room, heart rate (HR), blood pressure (BP), blood oxygen saturation (SpO_2_), bispectral index (BIS), and electrocardiography (ECG) were routinely monitored. The upper extremity venous access was established, and 6 L/min of pure oxygen was inhaled for 5 min. Before anesthesia induction, patients in DEX group were given continuous intravenous infusion of dexmedetomidine 0.4 *μ*g. kg-1. h-1 throughout the end of the anesthesia, and the NS group was given a continuous infusion of the same volume of normal saline simultaneously until the end of the anesthesia. Both groups were induced by intravenous injection of propofol 2-3 mg/kg, sufentanil 0.2-0.4 *μ*g/kg, and atracuramide cissilate 0.2 mg/kg.

#### 2.3.2. Maintenance of Anesthesia

After the tracheal intubation was connected to the ventilator, sevoflurane was used to maintain general anesthesia by continuous inhalation, and the end-expiratory concentration was maintained at 1.5% to 2%. At the same time, the dose of sufentanil was adjusted according to mean blood pressure (MBP), heart rate (HR), and bispectral index (BIS) values, and the additional dose was generally controlled at 0.1-0.3 *μ*g/kg, to maintain the BIS value at 45-60, and the addition was stopped 30 min before the end of the operation. According to the needs of the operation and the expected end time of the operation, atracuramide cissilate was added at a single additional dose of 0.1 mg/kg, and the addition was stopped 1 hour before the end of the operation. Intraoperative DEX group received dexmedetomidine maintenance dose of 0.4 *μ*g·kg-1. h-1 until the end of the operation. The NS group was infused with the same volume of normal saline until the end of the operation. At the end of the operation, the patients in both groups stopped inhaling sevoflurane, and the oxygen concentration was adjusted to 100%, at a flow rate of 6 L/min.

The article "Effects of Dexmedetomidine on Postoperative Pain and Recovery Time in Obese Patients" was retracted in 2023. Reasons: suspected computer-generated content; unreliable results or conclusions; concerns about the data; concerns about the results or conclusions.

#### 2.3.3. Recovery from General Anesthesia

After the operation, all patients were transferred to PACU with tracheal tube for mechanical ventilation and given sufentanil analgesia according to the patient's pain during operation. The patients in the DEX group continued to pump dexmedetomidine 0.2 *μ*g·kg-1. h-1 until the end of extubation, and the NS group was infused with the same volume of normal saline for the same time until the end of extubation. Then whether the patient conforms to the characteristics of extubation was observed, such as hemodynamic stability, spontaneous breathing, eye opening, consciousness recovery, and muscle strength recovery. After extubation, the patient's blood pressure, heart rate, respiration, and other vital signs were closely monitored until stable and then returned to the ward.

### 2.4. Outcomes

Anesthesia, surgery, postoperative extubation, and recovery time were recorded in the two groups of patients. The shorter the time, the better the sedative and analgesic effect of dexmedetomidine. Visual Analogue Scale (VAS) immediately 6 h, 12 h, and 24 h after the operation and the occurrence of adverse reactions were recorded. A straight line was divided into 9 equal parts, and the two ends represent 0 points of no pain and 10 points of severe pain, and the patients use a line to mark the value according to their subjective feelings to reflect the degree of pain. Measurements are required before and after treatment [6]. Adverse effects of anesthesia include nausea and vomiting, chills, agitation, and bradycardia.

### 2.5. Statistical Analysis

All indicate at each time point for the treatments were tested for normality using Shapiro–Wilk test. Since not all variables were normally distributed (*P* < 0.05), they were transformed by computing the log of the variable. SPSS 20.0 statistical software was used for data analysis. The measurement data conforming to the normal distribution were expressed as mean ± standard deviation (±s), and the *t* test was used for comparison between groups; the enumeration data was expressed as cases (%), and the *χ*2 test was used for comparison between groups. A *P* value of <0.05 was statistically significant.

The article "Effects of Dexmedetomidine on Postoperative Pain and Recovery Time in Obese Patients" was retracted in 2023. Reasons: suspected computer-generated content; unreliable results or conclusions; concerns about the data; concerns about the results or conclusions.

## 3. Results

### 3.1. Baseline Data

The DEX group (*n* = 50) included 31 males and 19 females. The average age was 31.53 ± 5.1 years old, the average body mass index (BMI) was 37.95 ± 1.52 kg/m^2^, and there were 30 cases of grade I, 15 grade II cases, and 5 grade III cases. The NS group (*n* = 50) included 33 males and 17 females. The mean age was 32.02 ± 5.33 years old, the mean body mass index (BMI) was 38.14 ± 1.31 kg/m^2^, and 33 cases were classified as I grade, 14 grade II cases, and 3 grade III cases. There was no significant difference in clinical data between the two groups (*P* > 0.05) as shown in Table 1.

### 3.2. Anesthesia Time, Operation Time, Postoperative Extubation, Recovery Time

Patients in the DEX group had considerably reduced anesthetic, operation, postoperative extubation, and recovery times than those in the NS group (*P* < 0.05) as shown in Table 2.

### 3.3. VAS Score

The VAS of the patients in the DEX group were significantly lower than those in the NS group immediately 6 h, 12 h, and 24 h after the surgery (*P* < 0.05) as shown in Table 3.

### 3.4. Adverse Reactions to Anesthesia

The adverse reactions of anesthesia in the two groups were observed, including nausea and vomiting, chills, restlessness, and bradycardia. The incidence of adverse reactions of anesthesia in the DEX group was significantly lower than that in the NS group (*P* < 0.05) as shown in Table 4.

## 4. Discussion

With the increasing number of obese people, “weight loss” has become a hot topic in terms of health and people's pursuit of beauty. Obesity is a metabolic disease that is associated with a variety of complications, including osteoarthritis or degenerative diseases, diabetes, hypertension, asthma, and sleep apnea syndrome. [9]. With economic development and changes in dietary structure, the number of obese people in China has increased significantly. Laparoscopic bariatric surgery is frequently used to treat obesity and metabolic disorders. As a result, anesthesia drugs and safety issues in the process of surgical treatment of obese patients has received increasing attention. However, obesity is associated with the circulatory system and respiratory system of patients and affects the distribution, systemic clearance, and plasma protein binding rate of narcotic drugs, so as to change the pharmacokinetics and pharmacodynamics of narcotic drugs, resulting in dismal postoperative pain relief outcome and surgical treatment [10]. Dexmedetomidine is a lipid-soluble drug with high protein binding rate, which can stabilize hemodynamics, reduce the excessive excitation of the sympathetic nervous system, and play an effective sedative and analgesic effect [11, 12]. More clinical studies have shown that dexmedetomidine also has antianxiety, lowering blood pressure, inhibiting salivary gland secretion, and diuretic effects [13].

The article "Effects of Dexmedetomidine on Postoperative Pain and Recovery Time in Obese Patients" was retracted in 2023. Reasons: suspected computer-generated content; unreliable results or conclusions; concerns about the data; concerns about the results or conclusions.

In this study, the two groups of patients were pumped with dexmedetomidine and normal saline, respectively. The results showed that the operation, anesthesia, postoperative extubation, and recovery time of patients in the dexmedetomidine group were significantly lower than those in the normal saline group; the VAS and the incidence of adverse reactions were significantly lower in the dexmedetomidine group than those in the normal saline group. This also demonstrates that dexmedetomidine can successfully decrease the recovery time of bariatric surgery in obese patients, minimize postoperative discomfort, and improve anesthetic resuscitation quality. [14]. Dexmedetomidine produces sedative and hypnotic effects by acting on the presynaptic or postsynaptic *α*2 adrenergic receptors in the nucleus locus coeruleus *α*2 in the brain. And can be awakened by external stimuli or language without affecting respiratory function [15, 16]. Moreover, it has analgesic effect on *α*2 receptors in the spinal cord and cooperates with inhaled anesthetics; opioid analgesics to produce good analgesia and the sedative effect can reduce the dosage of other anesthetics, analgesic, and hypnotic drugs and ensure the safety of anesthesia [17, 18]. The use of dexmedetomidine can improve the tolerance of obese patients to tracheal intubation, reduce postoperative agitation, and realize awake extubation, which is conducive to postoperative recovery after laparoscopic bariatric surgery.

Preoperative pumping of dexmedetomidine can promote stable induction of anesthesia, effectively suppress pain during propofol injection, and reduce the dose of other drugs, thereby reducing anesthesia side effects [19]. Continuous pumping of dexmedetomidine during the maintenance period of general anesthesia can maintain the hemodynamic stability of the patient, leading to a manageable maintenance period of anesthesia without affecting the recovery time of the patient [20]. This suggests that dexmedetomidine can maintain hemodynamic stability in surgical anesthesia in clinically obese patients, and the effects of different doses of dexmedetomidine are equivalent. The possible explanation is that after dexmedetomidine enters the human body, it can directly act on the locus coeruleus receptors in the brain, thereby exerting significant antianxiety, anti-irritability, and sedative effects, which in turn provides a favorable effect for the stability of the patient's hemodynamics [21, 22]. In addition, dexmedetomidine anesthesia helps reduce the patient's stress response. It might be attributed to the fact that dexmedetomidine is one of the highly selective *α*2 adrenergic receptor (*α*2AR) agonists, which mainly acts on the *α*2AR of the brain and spinal cord, thereby inhibiting neuronal discharge and the release of norepinephrine [23]. It further reduces the response of the sympathetic nervous system and finally exerts sedative, anxiolytic, and analgesic effects [24, 25]. It is concluded that 2 *μ*g/kg dexmedetomidine has favorable anesthesia effect in the operation of clinical obesity patients, can provide good analgesia and recovery quality, is conducive to reducing the degree of stress response of patients, and is associated with a lower risk of adverse events.

The article "Effects of Dexmedetomidine on Postoperative Pain and Recovery Time in Obese Patients" was retracted in 2023. Reasons: suspected computer-generated content; unreliable results or conclusions; concerns about the data; concerns about the results or conclusions.

This experiment is a randomized and controlled clinical study, which is controlled according to different doses, and the basic anesthesia methods are the same, which greatly reduces the impact on the controls. The results of this experiment show that the three groups of anesthesia methods can be safely used in the surgical treatment of clinical obesity patients, but preoperative application of loading dose of dexmedetomidine induction can significantly reduce the amount of intraoperative opioids, reduce extubation time and early postoperative agitation, improve perioperative hemodynamic stability and recovery quality of patients, reduce postoperative inflammatory response and the incidence of early postoperative POCD, improve perioperative safety, and facilitate early postoperative recovery of patients.

Although this study is only a traditional observational clinical study, no basic experiments and in vitro and in vivo experiments were conducted to explore how dexmedetomidine affects patients with obesity surgery, this study provides some ideas for the future treatment of the disease. The following limitations might undermine the results: (1) the overall sample size of this experiment is small, which may cause biased results. Future studies with larger sample size are required to reduce experimental bias. (2) This study only collected the effects of these three anesthesia methods on patients' early postoperative pain and extubation time and failed to conduct long-term postoperative follow-up. Subsequent studies are needed to extend the follow-up time to six months or one year, so as to accurately observe the effects of dexmedetomidine on long-term functional recovery after surgery in clinically obese patients. (3) This study failed to follow the double-blind principle in the recording of perioperative hemodynamic changes and postoperative follow-up.

The article "Effects of Dexmedetomidine on Postoperative Pain and Recovery Time in Obese Patients" was retracted in 2023. Reasons: suspected computer-generated content; unreliable results or conclusions; concerns about the data; concerns about the results or conclusions.

To sum up, the use of appropriate low-dose dexmedetomidine in the surgical treatment of clinical obesity patients can effectively shorten the recovery time of patients, reduce postoperative pain and adverse reactions, and improve the quality of general anesthesia recovery period. The drug can be safely used in the surgical treatment of obese patients and merits application in clinic setting.

## Figures and Tables

**Table 1:** Comparison of general data of the two groups of patients.

Groups	Gender		Age (year)	BMI (kg/m^2^)	ASA grade		
	Male	Female			I	II	III
DEX group (*n* = 50)	31	19	31.53 ± 5.1	37.95 ± 1.52	30	15	5
NS group (*n* = 50)	33	17	32.02 ± 5.33	38.14 ± 1.31	33	14	3
*t*	0.174		0.47	0.67	0.134		
*P*	0.677		0.639	0.504	0.714		

**Table 2:** Comparison of anesthesia, surgery, postoperative extubation, and recovery time between the two groups of patients [($\bar{\text{x}}\pm \text{s}$), min.].

Groups	Anesthesia time	Operation time	Postoperative extubation time	Wake up time
DEX group (*n* = 50)	122.5 ± 10.65	113.25 ± 4.77	148.64 ± 6.54	30.15 ± 2.95
NS group (*n* = 50)	127.37 ± 10.20	115.89 ± 3.91	161.26 ± 5.03	33.28 ± 3.14
*t*	2.335	3.027	10.816	5.137
*P*	0.022	0.003	0.001	0.001

**Table 3:** Comparison of VAS scores between the two groups of patients ($\bar{\text{x}}\pm \text{s}$).

Groups	Immediately after surgery	6 h after surgery	12 h after surgery	24 h after surgery
DEX group (*n* = 50)	1.46 ± 0.76	3.08 ± 0.68	2.23 ± 1.12	1.66 ± 0.24
NS group (*n* = 50)	1.80 ± 0.81	3.85 ± 0.73	2.95 ± 0.97	2.28 ± 0.35
*t*	2.165	5.458	3.436	10.33
*P*	0.033	0.001	0.001	0.001

**Table 4:** Comparison of the incidence of adverse reactions of anesthesia in the two groups of patients [*n* (%)].

Groups	Nausea and vomiting	Chills	Restless	Bradycardia	Total incidence
DEX group (*n* = 50)	2 (0.04)	1 (0.02)	0 (0)	0 (0)	3 (0.06)
NS group (*n* = 50)	5 (0.10)	3 (0.06)	2 (0.04)	0 (0)	10 (0.20)
*χ* ^2^	—	—	—	—	4.332
*P*	—	—	—	—	0.037

## Data Availability

All data generated or analysed during this study are included in this published article.
